RETRACTED

# LncRNA LINC01305 silencing inhibits cell epithelial‐mesenchymal transition in cervical cancer by inhibiting TNXB‐mediated PI3K/Akt signalling pathway

**DOI:** 10.1111/jcmm.14161

**Published:** 2019-01-29

**Authors:** Shu‐Ping Yan, Dan‐Xia Chu, Hai‐Feng Qiu, Ya Xie, Chun‐Fang Wang, Jian‐Ying Zhang, Wen‐Cai Li, Rui‐Xia Guo

**Affiliations:** ^1^ Department of Pathology The First Affiliated Hospital of Zhengzhou University Zhengzhou Henan Province P.R. China; ^2^ Department of Gynecology The First Affiliated Hospital of Zhengzhou University Zhengzhou Henan Province P.R. China; ^3^ Institute of Medical and Pharmaceutical Sciences, Zhengzhou University Zhengzhou Henan Province P.R. China; ^4^ Department of Pathology School of Basic Medicine, Zhengzhou University Zhengzhou Henan Province P.R. China; ^5^ Henan Key Laboratory for Tumor Pathology Zhengzhou Henan Province P.R. China

**Keywords:** cervical cancer, epithelial‐mesenchymal transition, invasion, long non‐coding RNA LINC01305, migration, PI3K/Akt signalling pathway, TNXB

## Abstract

Cervical cancer (CC) remains one of the leading malignancies afflicting females worldwide, with its aetiology associated with long‐term papillomavirus infection. Recent studies have shifted their focus and research attention to the relationship between long non‐coding RNAs (lncRNAs) and CC therapeutic. Thus, the aim of the current study was to investigate the underlying mechanism of lncRNA LINC01305 on the cell invasion, migration and epithelial‐mesenchymal transition (EMT) of CC cells via modulation of the PI3K/Akt signalling pathway by targeting tenascin‐X B (TNXB). The expressions of LINC01305, TNXB, MMP2, MMP9, E‐cadherin, vimentin, PI3K, Akt, p‐PI3K, p‐Akt and TNXB were detected in this study. After which, the cell invasion and migration abilities of the CC cells were determined respectively. Bioinformatics and the application of a dual luciferase reporter gene assay provided verification indicating that TNXB is the target gene of lncRNA LINC01305. Reverse transcription quantitative polymerase chain reaction (RT‐qPCR) and western blot analysis methods revealed that the expressions of MMP2, MMP9, vimentin, PI3K, Akt, p‐PI3K and p‐Akt were decreased following the down‐regulation of LncRNA LINC01305 or overexpression of TNXB. LncRNA LINC01305 silencing or TNXB overexpression was noted to decrease the migration and invasion of SiHa cells. Taken together, the key findings of the current study present evidence suggesting that lncRNA LINC01305 silencing suppresses EMT, invasion and migration via repressing the PI3K/Akt signalling pathway by means of targeting TNXB in CC cells, which ultimately provides novel insight and identification of potential therapeutic targets for CC.

RETRACTED

## 1 INTRODUCTION

Cervical cancer (CC) remains secondary only to breast cancer as the foremost malignancy afflicting females on a global scale.^1^ Pertinent risk factors are comprised of genetic susceptibility, viral infection and environmental factors all are related to the aetiology of CC.^2^ Owing to improved cytological screening and DNA testing methods, the incidence of CC has remarkably decreased in developed countries; nevertheless, for those without access to health care across the world, CC continues to be a major stumbling block, with studies reporting there to be approximately 250 000 deaths and 500 000 new cases on an annual basis.^3^, ^4^ Persistent papillomavirus infection has been identified as the leading cause of CC with human papillomavirus (HPV) detected in approximately 99% of CC, in particular the oncogenic subtypes HPV18 and 16.^5^ A recent study concluded that epithelial‐mesenchymal transition (EMT) plays a critical role in the progression of CC.^6^ At present, patients with early‐stage and locally advanced CC tumours are often treated by means of radical therapy, chemotherapy or combination therapy, while those with recurrent and persistent disease have limited treatment options.^1^, ^7^ Therefore, it is necessary to do deeper investigations in an attempt to identify novel CC treatment approaches based on the molecular mechanisms that facilitate the development and progression of CC.^8^

Long non‐coding RNAs (lncRNAs) are defined as genomic transcriptions that are longer than 200 nucleotides (nt) that do not possess protein coding capability due to a lack of an open reading frame of a required length.^9^ Various studies have implicated lncRNAs to the biological mechanisms observed in cancer and highlighted their potential as biomarkers and therapeutic targets.^10^ A number of lncRNAs have been shown to play significant roles in the pathogenesis of several cancers including colorectal, kidney and breast cancers.^11^, ^12^, ^13^ By means of analysis of the bioinformatics prediction website for the CC microarray expression profile data, lncRNA LINC01305 was identified as the most notably overexpressed lncRNAs (GSE63514). Tenascin‐X (TNX) is a significant member (450 kDa) of the tenascin family of extracellular matrix glycoproteins and its deficiency in mice and human has been correlated to a diverse group of connective tissue disorders, affecting the skin, joints and vessels.^14^ The TNX gene is composed of TNXA and TNXB, and TNXB embraces epidermal growth factor, series of heptad, a signal peptide and fibronectin type III repeats, as well as a fibrinogen globe and a serine‐proline‐rich domain.^14^, ^15^ Phosphoinositide 3‐kinase (PI3K) serves as a heterodimeric protein, consisting of a regulatory subunit (p85a/b) and a catalytic submit (p110a/b/g/d). Activated PI3K in addition to its downstream target Akt/PKB can regulate cell proliferation, apoptosis and oncogenesis, as well as critical signalling molecules and key survival factors.^16^ Lu et  al asserted that the inhibited expression of lncRNA (highly up‐regulated in liver cancer) HULC could drastically suppress chronic myeloid leukaemia cell proliferation and promote apoptosis partially through inactivation of the PI3K/Akt signalling pathway by repressing its phosphorylation.^17^ Hence, based on the aforementioned exploration of literature, the present study aims to confirm the hypothesis that lncRNA LINC01305 silencing might suppress EMT, invasion and migration via repressing the TNXB‐mediated PI3K/Akt signalling pathway in CC cells.

RETRACTED

## 2 MATERIALS AND METHODS

### 2.1 Cell culture

Cervical cancer cell lines SiHa, Hela, C‐33A, Ca ski, ME‐180, MS751 (purchased from the Cell Bank of the Chinese Academy of Sciences, Shanghai, China) were cultivated by the Roswell Park Memorial Institute‐1640 (RPMI‐1640) medium containing 10% foetal bovine serum (FBS) (100 U/mL penicillin and 100 μg/mL streptomycin) (PeproTech Inc, Rocky Hill, NJ) in an incubator at 37°C with 5% CO_2_ until the cells grew to the logarithmic phase.

### 2.2 Target gene prediction by bioinformatics and verification

Cervical cancer microarray expression profile data (GSE63514) as well as the relevant microarray probe set annotation were downloaded from gene expression omnibus (GEO) database (http://www.ncbi.nlm.nih.gov/geo). The two aforementioned microarrays were detected by Affymetrix Human Genome U133 Plus 2.0 Array and Agilent‐062918 OE Human lncRNA Microarray V4.0 028004. The microarray database underwent background correction and normalization through the Affy of r software, after which^18^ linear models‐empirical Bayes statistical methods and conventional *t* test methods were applied to construct the non‐specific filtration of expression profile data, in order to screen out the differentially expressed lncRNAs.^19^ Multi Experiment Matrix website (MEM, http://biit.cs.ut.ee/mem/) was employed to predict the differentially expressed lncRNAs, and the Database for Annotation, Visualization and Integrated Discovery (DAVID) (https://david.ncifcrf.gov/) to undergo Kyoto Encyclopedia of Genes and Genomes (KEGG) analysis of the target gene to identify co‐expression genes.

The wild‐type (wt) 3ʹ‐untranslated region (UTR) and mutant (mut) 3ʹ‐UTR of TNXB were amplified, while the primer sequence was prepared by Shanghai Sangon biological Engineering Technology & Services Co., Ltd. (Shanghai, China). The TNXB was released by restriction with XhoI and NotI enzyme digestion and ligated into psi‐Cpsi‐CHECK‐2 vector (Promega Corp., Madison, Wisconsin) by using T4 DNA ligase to obtain TNXB‐wt and TNXB‐mut plasmids. A total of 200 μmol/L empty vector plasmid as negative control (NC) or LINC01305, 100 ng plasmid (TNXB‐wt or TNXB‐mut), after mixture and incubation with 50 μL RiboFECTTMCP buffer and 5 μL transfection reagents, co‐transfection with SiHa cells were performed in accordance with the instructions of RiboFECTTMCP transfection kit (Guangzhou RiboBio Co., Ltd., China). SiHa cells with a density of 5 × 10^4^ cells/well were subsequently cultured in a 24‐well plate for 48 hours, and lysed in order to determine luciferase activity. Each group was set up with three parallel wells with a blank control, with each experiment repeated three times. In accordance with the instructions of dual luciferase reporter gene assay kit (RG005; Beyotime biotechnology Co., Shanghai, China), the cells were rinsed with phosphate buffer solution (PBS) and lysed with 200 μL lysate for 15 minutes. Firefly luciferase reporter gene assay kit (RG005; Beyotime biotechnology Co.) and a microplate reader (MK3, Thermo fisher scientific Inc, Waltham, MA) were then employed to examine luciferase activity at 560 nm.

RETRACTED

### 2.3 RNA immunoprecipitation assay

SiHa cells (2 × 10^7^) were selected and treated according to Magna RNA immunoprecipitation (RIP) TM RNA‐Binding Protein Immunoprecipitation Kit (Millipore Corp., Billerica, MA, USA). The cells were then added with 5 μg rabbit anti‐human AGO2 antibody and normal rabbit anti‐immunoglobulin G (IgG) antibody, incubated in cell lysate overnight at 4°C while rotated. The protein‐RNA complex was collected following the acquisition of the specific protein from the cells with 2 μg specific TNXB antibody (sc‐271594; Santa Cruz Biotechnology, Inc, Santa Cruz, CA, USA). Proteinase K was subsequently used to remove the proteins and extract the RNA molecules. During the experiment, RIP washing buffer was used to wash the magnetic beads in a repetitive manner in order to eradicate non‐specific adsorption as much as possible. RNA molecules were subsequently obtained by means of reverse RT‐qPCR.

### 2.4 Subcellular localization prediction and identification

The subcellular localization of LINC01305 in SiHa cells was predicted in connection with the bioinformatics prediction website http://lncatlas.crg.eu/ and verified by fluorescence in situ hybridization (FISH). Oligonucleotide probe (Downers Grove, IL, USA) marked by Cy5 was designed for LINC01305, with the specific procedures applied as follows: SiHa cells were seeded into a six‐well plate with a cover glass and then placed into a sterile cover glass to facilitate cell growth on the cover glasses. After the cells had been cultured for 1 hour and reached 70% confluence, the culture medium was removed and the glass was taken out and rinsed twice with PBS. The cells were then fixed using 1 mL 4% paraformaldehyde, cultured with 1 mL proteinase K (2 μg/mL) and 1 mL glycine at room temperature for 5 minutes respectively, after which, the cells were rinsed twice with phosphate buffered saline + Tween 20 (PBST). The cells were then cultured with 1 mL acetylation reagent for 10 minutes, rinsed three times with PBST and incubated with 250 μL prehybridization solution at 42°C for 1 hour. After that, the prehybridization solution was collected and added with 250 μL hybridization solution containing probe (300 ng/mL) at 42°C overnight. The hybridization solution was collected and reacted with 50% formamide, 2× SSC, 0.1% NP‐40 and 70% ethanol in sequence at 42°C for 10 minutes; after three PBST rinses, the solution was sealed with 1 mL 3% bull serum albumin (BSA) for 1 hour. The antibody was diluted by 3% BSA with the final concentration of 20 μg/mL, added onto the cover glass and then incubated for 5 hours under conditions void of light. The glass was subsequently rinsed three times (3 minutes each time). Diamidino‐phenylindole (DAPI) (1:800) was diluted using PBST, and added into a 24‐well plate and stained for 5 minutes. After the plate had been rinsed three times (3 minutes each time) it was sealed with anti‐fluorescence quenching agent. Five different visual fields were observed and photographed under a fluorescence microscope (400×; Olympus optical Co., Ltd, Tokyo, Japan).

RETRACTED

### 2.5 Construction of expression vector

Trizol (Invitrogen Inc, Carlsbad, CA, USA) was subsequently applied in order to extract the total RNA of the SiHa cells, cDNA synthesis kit (Fermentas Inc, Hanover, MD, USA) was used to synthesize cDNA of LINC01305 and Hind III and BamH I restriction site to artificially synthesize the primer of LINC01305. The double enzyme method was used to cut the purified products of PCR and linked with pcDNA3.1 (+) plasmid in order to construct the pcDNA3.1‐LINC01305‐overexpressed recombinant plasmid.^20^ The interference RNA sequence and control sequence of LINC01305 gene were synthesized by Shanghai GenePharma Co., Ltd. (Shanghai, China) based on pSH‐U6‐GFP plasmid (Vigenebio, Genecopoeia, Rockville, MD, USA).

### 2.6 Cell transfection and grouping

SiHa, Hela, C‐33A, Ca ski, ME‐180 and MS751 cells at the logarithmic phase were normally douched and treated by 0.05% trypsin (Dingguo Biological Reagent, Co., Ltd., Beijing, China) in order to prepare single cell suspension. The cells were adjusted to a concentration of 3 × 10^4^ cells/mL and seeded into a T25 culture bottle. After 24 hours of cell adherence, the culture medium was removed. Lipofectamine 2000 transfection reagent (Invitrogen Inc) was used to transfect the cells, which were then randomly assigned into seven groups namely: the blank (without transfection), LINC01305‐negative control (NC) (transfected with empty vector pcDNA3.1 (+) plasmid), LINC01305 (transfected with LINC01305 overexpressed plasmid), siRNA‐NC (transfected with empty vector pSH‐U6‐GFP plasmid), siRNA‐LINC01305 (transfected with siRNA‐LINC01305 plasmid), siRNA‐TNXB (transfected with siRNA‐TNXB plasmid) and siRNA‐LINC01305 + siRNA‐TNXB (transfected with siRNA‐LINC01305 plasmid and siRNA‐TNXB plasmid) groups. With the use of sterile (eppendorf) EP tube, lipofectamine 2000 and plasmid DNA were prepared: 5 µL lipofectamine 2000 + 100 µL serum‐free medium was placed at room temperature for 5 minutes; 50 nmol/L plasmid DNA + 100 µL serum‐free medium was placed at room temperature for 20 minutes to form the complex of DNA and Liposome; serum‐free medium was used to wash the cells in the culture bottle. Serum‐free medium (without antibody) was added to the complex, mixed in a moderate fashion and added to the cells for transfection purposes. After transfection, the cells were cultured in a successive manner in an incubator at 37°C for 6 hours and in RPMI 1640 medium for 48 hours. Following the conclusion of the experiment, RT‐qPCR methods were applied to detect the expressions of LINC01305 and TNXB mRNA from the various cell samples among different cells. The cells exhibiting the most significant changes were selected for further detection and experimentation.

### 2.7 Reverse transcription quantitative **PCR**

The total RNA of each group was extracted by Trizol (Invitrogen Inc) and absorbance (A) value in each group at 260 and 280 nm (A_260_/A_280_) was measured. The ratio was set between 1.8 and 2.0. With VeriQuest™ SYBRTM Green One‐Step RT‐qPCR Master Mix kit (75705200RXN; Sigma‐Aldrich Chemical Company, St. Louis, MO, USA), 1 µL RNA was taken out from each group and used in reaction. The reaction conditions were conducted as follows: one cycle of cDNA synthesis at 50°C for 10 minutes, at 95°C for 10 minutes; 35‐45 cycles at 95°C for 15 seconds, at 60°C for 30 seconds. The reaction system was as follows: 25 µL VerQuest SYBR Green One‐Step RT‐qPCR Master Mix (2×), 0.5 µL Veri Quest 100× RT Enzyme Mix for SYBR Green Assay, 2.5 µL Forward Primer (10 µmol/L), 2.5 µL Reverse Primer (10 µmol/L), 1 µL Template RNA and moderate diethyl pyrocarbonate (DEPC)‐treated RNase free water to make the reaction system up to 50 µL. The primer of LINC01305 was designed by Oligo7 software and the primers (Table 1) of TNXB and glyceraldehyde phosphate dehydrogenase (GAPDH) were obtained from https://pga.mgh.harvard.edu/primerbank/index.html. A solubility curve was constructed and used to assess the reliability of the obtained PCR results. The CT (threshold cycle) value was determined based on the following formula ∆Ct = CT_(target gene)_ − CT_(internal reference)_, ∆∆Ct = ∆Ct_(the experiment group)_ − ∆Ct_(the control group)_. The 2^−ΔΔCt^ was regarded as the relevant expression of the target gene in each group.^21^ Each experiment was repeated three times, with the average value subsequently obtained.

RETRACTED

**Table 1:** The primer sequences of RT‐qPCR

Gene	Forward primer (5ʹ‐3ʹ)	Reverse primer (5ʹ‐3ʹ)
LINC01305	CCACGCAGCTCTCCAACACTC	TTTGGGCGACTACAGAATCCA
TNXB	GTGGTCCAGTATGAGGACACG	CTGGTGGTCACGTCAGTCAC
GAPDH	CAGGGCTGCTTTTAACTCTGGTAA	GGGTGGAATCATATTGGAACATGT

Notes:

GAPDH, glyceraldehyde phosphate dehydrogenase; RT‐qPCR, reverse transcription quantitative polymerase chain reaction; TNXB, Tenascin‐X B.

### 2.8 Western blot analysis

Western blot analysis was applied in order to measure the protein expressions of migration‐related proteins (matrix metalloproteinase 2 [MMP2], matrix metalloproteinase 9 [MMP9]), epithelial cell marker protein (E‐cadherin) and mesenchymal cell marker protein (vimentin) and pathway‐related proteins (PI3K, Akt, p‐PI3K, p‐Akt, TNXB). Cells in each group were lysed by radioimmunoprecipitation assay (RIPA) lysis (Beyotime biotechnology Co.) and rinsed three times using pre‐cooled PBS. The cells were scraped down in a systematic manner and the samples were moved into a 1.5 mL centrifuge tube, and mixed thoroughly for complete lysis using the top end of an aspirator. Then, 14 000 *g* cell samples were centrifuged for 10 minutes and the supernatant was stored in −20°C conditions. The samples were persisted with the following steps of the experiment. Bicinchoninic acid (BCA) reagent kit (MultiSciences biotech Co, Ltd, Hangzhou, China) was used for quantifying protein expressions, and then samples were added with buffer solution and boiled at 95°C for 10 minutes. After that, samples underwent gel electrophoresis (the concentration of the gel was prepared based on the molecular weight of the protein). After the electrophoretic separation using polyacrylamide gel, protein was transferred onto a nitrocellulose membrane and sealed with 5% BSA for 1 hour. The primary antibody was then incubated at 4°C overnight. The primary antibody includes rabbit polyclonal antibody MMP2 (ab37150, 2 µg/mL), MMP9 (ab137867, 1:1000), E‐cadherin (ab40772, 1:1000), vimentin (ab16700, 1:100), PI3K (ab151549, 1:500), Akt (ab8805, 1:500), p‐PI3K (ab182651, 1:1000), p‐Akt (ab 8449, 1:500), mouse antibody TNXB (ab 67586, 1:500) and mouse antibody GAPDH (ab8245, 1:1000). After incubation of the primary antibody, the membrane was douched in 1× (Tris Buffer Solution+Tween) TBST solution and shaken three times using a shaking table (5 minutes each time). Next, the second antibodies of the mouse anti‐rabbit (Santa Cruz, CA, USA) or rabbit antimouse (Santa Cruz, CA) were added and incubated at room temperature for 2 hours, and rinsed three times using TBST (20 minutes each time). Enhanced chemiluminescence (ECL) was employed for development purposes. SmartView Pro 2000 (UVCI‐2100; Major Science, Co., Ltd., CA, USA) was used for photography, while Quantity One software was used for the gray value analysis of the protein bands.

RETRACTED

### 2.9 Scratch test

After 48 hours of transfection in each group, cell culture was continued until cell density was confirmed to have reached 80%‐90%. Scratches were made by a 200 μL middle‐size pipette along a ruler in a vertical fashion to the transverse line as far as possible. The cells were rinsed three times in order to remove the redundant cells following the addition of RPMI 1640 culture medium containing 10% FBS, which were cultured at 37°C in an incubator with 5% CO_2_. At 0 and 48 hours, cells were observed and photographed under an inverted phase contrast microscope (100×; Olympus Optical Co., Ltd). The scratch healing was dynamically viewed with the widths of each scratch among each group compared. The migration rate was calculated based on the following formula: scratch width at 48 hours/scratch width at 0 hour × 100%.

### 2.10 Transwell assay

Based on the Costar 24‐Well Transwell^TM^ instructions, a Transwell assay was conducted (Millipore Corp.). The Matrigel was stored at −20°C (Becton, Dickinson and Company, Bioscience, San Jose, CA, USA) and pre‐cooled at 4°C overnight for liquidation and diluted by serum‐free medium on ice in 1:1 dilution. The mixture was then added to the Transwell chamber (Costar, Cambridge, MA, USA) with 15 μL in each well and cultured at 37°C for 1 hour, and then rinsed three times using serum‐free medium for later use. The SiHa cells were digested and rinsed twice using serum‐free medium, with the number of cells recorded. The cell suspension (containing 1 × 10^5^ cells) was added to the apical chamber while serum‐free Dulbecco's Modified Eagle Medium (DMEM) was added for dilution of the cell suspension to 400 μL. Each group was ordered with three parallel wells. The basolateral chamber was added with 600 μL DMEM complete medium containing 15% FBS and incubated at 37°C with 5% CO_2_ over a period of 24 hours. After removal of the liquid in chambers, the cells on the surface of the basolateral chamber were removed with a cotton swab. The chambers were then immersed in stationary liquid (50% methyl alcohol) for 15 minutes and rinsed three times with PBS. Crystal violet staining was performed for 30 minutes, after which the chambers were dried. Six visual fields from each culture well were randomly selected, observed and photographed under an inverted microscope (200×, Olympus Optical Co., Ltd.), with the average number of cells in each view calculated accordingly.

RETRACTED

### 2.11 Statistical analysis

SPSS21.0 (IBM Corp., Armonk, NY, USA) software was employed for statistical analysis. Measurement data were expressed as mean ± SD, while *t *test methods were utilized for comparison between two groups, with one‐way ANOVA used for comparison among multiple groups. Enumeration data were presented as percentage and compared using a chi‐squared test. Comparison of enumeration data among multiple groups was performed by ANOVA and homogeneity test of variance; in the event variance values were significantly different, *q* test methods were applied for comparison between two groups; when variance was determined to be irregular, non‐parametric rank sum test was employed for inspection, and the inspection level *α* = 0.05, *P < *0.05 was considered to be statistically significant.

## 3 RESULTS

### 3.1 TNXB is a target gene of lncRNA LINCRNA01305

The analysis of the bioinformatics prediction website for the CC microarray expression profile data (GSE63514, Figure 1A), provided verification that lncRNA LINC01305 was the most significantly overexpressed lncRNAs. The MEM website was utilized to further confirm that TNXB was indeed the target gene of LINC01305 (Figure 1C) in addition to elucidating its involvement in the PI3K/Akt signalling pathway (Figure 1B). Compared with the TNXB‐wt and NC co‐transfection group, the luciferase activity in the TNXB‐wt and LINC01305 co‐transfection group apparently decreased (*P < *0.05). In comparison to the TNXB‐mut and NC co‐transfection group, there was no obvious difference detected in the TNXB‐mut and NC co‐transfection group (*P* > 0.05) (Figure 1D). The results obtained provided evidence indicating the existence of a target relationship between LINC01305 and the 3ʹ‐UTR of TNXB, which was further verified by RIP assay (Figure 1E).

**Figure 1:** TNXB is the target gene of lncRNA LINCRNA. A, The thermal image analysis of GSE63514. B, The prediction of the target gene of LINC01305 detected by bioinformatics website. C, The prediction of the biding site of LINC01305 and TNXB. D, The relative luciferase activity in each group; the experiments were analysed by independent sample *t* test. E, Results of binding site between LINC01305 and TNXB by RIP assay. *P < 0.05, compared with the co‐transfection group of TNXB‐wt and NC. lncRNA LINC01305, long non‐coding RNA LINC01305; TNXB, Tenascin‐X B; NC, negative control; RIP, RNA immunoprecipitation

RETRACTED

### 3.2 LncRNA LINCRNA is located in nucleus of SiHa cells

The bioinformatics prediction website http://lncatlas.crg.eu provided evidence indicating that the subcellular localization of LINC01305 was in nucleus (Figure 2A). The FISH method (Figure 2B) was applied to predict the subcellular localization of LINC01305 in SiHa cells. The green fluorescence was considered to be reflective of the distribution of LINC01305 in cells; the nucleus was stained blue by DAPI; while the merger of the former two figures provided indication that LINC01305 was mainly distributed in nucleus of the SiHa cells.

**Figure 2:** LncRNA LINCRNA is located in nucleus of SiHa cells. A, Prediction of LINC01305 subcellular localization in different cells through lncatlas.crg analysis. B, Verification of LINC01305 subcellular localization in SiHa cells (×400) whereby the nucleus was represented by blue, green represented the fluorescence localization of LINC01305, and the ruler = 25 μm. lncRNA LINC01305, long non‐coding RNA LINC01305; DAPI, Diamidino‐phenylindole

### 3.3 SiHa, Hela and C‐33A cell lines exhibit up‐regulated levels of LINC01305 but down‐regulated TNXB expressions

In order to select the CC cell lines with the optimal efficiency for the further experimentation, RT‐qPCR measures were employed to determine the expressions of LINC01305 and TNXB in SiHa, Hela, C‐33A, Ca ski, ME‐180 and MS751 cell lines (Figure 3). The results obtained indicated that when compared to the MS751 cells, the expressions of LINC01305 and TNXB among the ME‐180 cells exhibited no significant difference; the expression of LINC01305 in the SiHa, Hela, C‐33A and Ca ski cells was significantly elevated while that of TNXB was decreased; the expression of LINC01305 and TNXB in the SiHa, Hela and C‐33A did not exhibit any significant difference. Thus, based on the above results, we selected the SiHa, Hela and C‐33A cell lines for transfection.

**Figure 3:** SiHa, Hela and C‐33A cell lines exhibit up‐regulated LINC01305 but down‐regulated TNXB expressions. Data were expressed as mean ± SD (n = 3), and compared using one‐way ANOVA. *P < 0.05 compared with MS751 cells. #compared with Ca ski cells

### 3.4 LncRNA LINC01305 silencing increases TNXB mRNA expression

In order to investigate the role of LINC01305 and DLG2 in CC, varying expressions of LINC01305 and TNXB were introduced to the CC cells and followed by RT‐qPCR detection. The results obtained indicated that the expressions of LINC01305 and TNXB among the SiHa, Hela and C‐33A cell lines in each transfection group using RT‐qPCR methods, which are illustrated Figure 4. Compared with the blank group, the expressions of LINC01305 and TNXB in the LINC01305‐NC and siRNA‐NC groups showed no obvious difference (*P* > 0.05); LINC01305 expression was reduced while the TNCB expression exhibited no distinct difference in the siRNA‐LINC01305 + siRNA‐TNXB group; in the LINC01305 group, LINC01305 was markedly up‐regulated while TNXB was down‐regulated (*P* < 0.05); the siRNA‐LINC01305 group attenuated LINC01305 expression but increased TNXB expression (*P < *0.05); in the siRNA‐TNXB group, LINC01305 expression showed no difference and TNXB expression was reduced (*P* < 0.05). Among these three types of cell lines, the expressions of LINC01305 and TNXB in SiHa cells displayed the most statistically significant difference; hence, the SiHa cell line was selected for further experiments. These findings provided evidence that LncRNA LINC01305 silencing decreases the mRNA expression of TNXB*.*

RETRACTED

**Figure 4:** Expressions of TNXB was up‐regulated due to LncRNA LINC01305 silencing. Expressions of genes in SiHa, Hela and C‐33A were expressed as mean ± SD (n = 3), and compared using one‐way ANOVA. *P < 0.05 compared with the blank group, RT‐qPCR, reverse transcription quantitative polymerase chain reaction. TNXB, Tenascin‐X B; NC, negative control

### 3.5 LncRNA LINC01305 silencing reduces protein expressions of MMP2, MMP9, vimentin, p‐PI3K and p‐Akt but increases those of E‐cadherin and TNXB in SiHa cells

To further explore the role of LINC01305 and TNXB in MMPs, EMT and PI3K/Akt signalling pathway, the protein expressions of MMP2, MMP9, E‐cadherin, vimentin, PI3K, Akt, p‐PI3K, p‐Akt and TNXB in each group were examined by western blot analysis means, the results of which are depicted in Figure 5. The protein expressions of PI3K and Akt displayed no distinct difference among the SiHa cells of each group (all *P* > 0.05). In comparison to the blank group, the protein expressions of MMP2, MMP9, E‐cadherin, vimentin, p‐PI3K, p‐Akt and TNXB displayed no notable difference in the LINC01305‐NC, siRNA‐NC and siRNA‐LINC01305 + siRNA‐TNXB groups (all *P* > 0.05); while the protein expressions of MMP2, MMP9, vimentin, p‐PI3K and p‐Akt were noted to have been remarkably enhanced, while those of E‐cadherin and TNXB were notably diminished in the LINC01305 group (all *P* < 0.05). A contrasting trend was observed in relation to the tendencies of the siRNA‐LINC01305 group (all *P < *0.05). In comparison with the siRNA‐TNXB group, the siRNA‐LINC01305 + siRNA‐TNXB group decreased protein expressions of MMP2, MMP9, vimentin, p‐PI3K and p‐Akt were detected, while elevated levels of E‐cadherin and TNXB were observed (all *P* < 0.05). The results obtained indicated that, LncRNA LINC01305 silencing down‐regulates the protein expressions of MMP2, MMP9, vimentin, p‐PI3K, p‐Akt and TNXB in SiHa cells.

RETRACTED

**Figure 5:** Protein expressions of MMP2, MMP9, vimentin, p‐PI3K and p‐Akt were reduced while E‐cadherin and TNXB protein expressions elevated owing to LncRNA LINC01305 silencing. A, The protein expressions of MMP2, MMP9, E‐cadherin, vimentin, PI3K, Akt, p‐PI3K, p‐Akt and TNXB in SiHa determined by western blot analysis, expressed as mean ± SD (n = 3), in which *x*‐axis represented different proteins in each group, and *y*‐axis represented relative protein expressions (the gray values of target bands to internal control bands). B, The electrophoresis bands of MMP2, MMP9, E‐cadherin, vimentin, PI3K, Akt, p‐PI3K, p‐Akt and TNXB proteins in SiHa cells. *P < 0.05 compared with the blank group. #*P* < 0.05, compared with siRNA‐TNXB group. MMP2, matrix metalloprotease 2; MMP9, matrix metalloprotease 9; p‐PI3K, phospho‐phosphatidylinositol 3‐kinase; p‐Akt, phospho‐protein kinase b; TNXB, Tenascin‐X B; NC, negative control

### 3.6 LncRNA LINC01305 silencing decreases cell migration of SiHa cells

Next, a scratch test was applied to measure the effect of LINC01305 on the cell migration of the SiHa cells, the results obtained are illustrated in Figure 6. When compared with the blank group, cell migration of the SiHa cells exhibited no notable difference in the LINC01305‐NC and siRNA‐NC groups (both *P* > 0.05), while strengthened rates were detected in both the LINC01305 group and siRNA‐TNXB group (*P* < 0.05), with weakened rates detected in the siRNA‐LINC01305 group (both *P* < 0.05). In comparison with the siRNA‐TNXB group, the siRNA‐LINC01305 + siRNA‐TNXB group had diminished rates of SiHa cellular migration (*P* < 0.05). Based on these results, we asserted that LncRNA LINC01305 silencing decreases the cell migration of SiHa cells.

**Figure 6:** LncRNA LINC01305 silencing declined cell migration in SiHa cells. A, The images of scratch healing of SiHa cells in each group (100×), in which the ruler = 100 μm. B, The percentage of cell migration width of SiHa cells in each group expressed as mean ± SD (n = 3), in which *x*‐axis represented different groups, and *y*‐axis represented scratch healing percentage. *P < 0.05 compared with the blank group. #*P* < 0.05 compared with the siRNA‐TNXB group. TNXB, Tenascin‐X B; NC, negative control

RETRACTED

### 3.7 LncRNA LINC01305 silencing reduces cell invasion of SiHa cells

Transwell assay was employed to assess cell invasion in each group (observed and counted under an inverted microscope (200×) (Figure 7). In comparison to the blank group, the cell inversion in the LINC01305‐NC and siRNA‐NC groups displayed no distinct difference (both *P* > 0.05), while enhancements were detected in the LINC01305 group and siRNA‐TNXB group, with decreases observed in the siRNA‐LINC01305 group (both *P* < 0.05). When compared with the siRNA‐TNXB group, the siRNA‐LINC01305 + siRNA‐TNXB group displayed attenuated SiHa cell migration (*P* < 0.05). These results suggested that LncRNA LINC01305 silencing could act to reduce the cell invasion of SiHa cells.

**Figure 7:** LncRNA LINC01305 silencing reduces cell invasion in SiHa cells. A, The images of transwell invasion of SiHa cells in each group (200×), in which the ruler = 50 μm. B, The number of cell invasion of SiHa cells in each group expressed as mean ± SD (n = 3), in which *x*‐axis represented different groups, and *y*‐axis represented the number of cells that penetrating the Transwell chamber covered with Matrigel. *P < 0.05 compared with the blank group. #*P* < 0.05 compared with the siRNA‐TNXB group. TNXB, Tenascin‐X B; NC, negative control

## 4 DISCUSSION

Significant existing literature has provided verification indicating the involvement of lncRNAs in cancer biology, with lncRNAs exhibiting stimulated levels in a variety of malignancies, highlighting their usefulness as biomarkers and therapeutic targets.^10^, ^22^, ^23^ Thus, the present study aimed to explore the effects of the novel lncRNA LINC01305 on the cell invasion, migration and EMT of CC through the PI3K/Akt signalling pathway by targeting TNXB. A key observation of the current study revealed that specific knockdown of lncRNA LINC01305 expression inhibited the PIK/Akt signalling pathway by targeting TNXB, which ultimately suppressed EMT, cell invasion and migration of CC.

Initially, in connection with a microarray‐based gene expression analysis, we asserted the hypothesis that there was a target relationship between LINC01305 and TNXB, and that LINC01305 targeted TNXB through the regulation of the PI3K‐Akt signalling pathway in CC. The in vitro experiment subsequently provided verification indicating that TNXB was negatively regulated by LINC01305 through activation of the PI3K‐Akt signalling pathway. Moreover, the lncRNA LINC01305 was noted to be overexpressed while TNXB was under‐expressed in CC cells, which provided further evidence in regard to the prediction results as well as the results of the in vitro experiment. A previous study investigated the lncRNA regulation of transcriptional or post‐transcriptional gene and demonstrated that some interactions between altered lncRNA function and gene expression have been involved in clinical disease phenotypes,^24^ and concluded by highlighting the significance of lncRNA‐mediated regulatory networks. Recently, accumulating lncRNAs have been implicated in the progression of CC, including lncRNA HOTAIR, lncRNA MALAT1, lncRNA LET and lncRNA CCAT2.^25^, ^26^, ^27^, ^28^ Existing literature has revealed that lncRNAs play a role in CC through the regulation of various signalling pathways. ANRIL has been correlated with poor CC prognoses and play crucial roles in the process of tumourigenesis through activation of the PI3K‐Akt signalling pathway.^29^ The aforementioned study further highlighted that the activation of the PI3K‐Akt signalling pathway is accompanied by deterioration in the condition of CC patients, which was consistent with the observations of our study. As early as the year 1999, saw reports earmark TNX as a potential biomarker owing to its role as a biological defender in cases of CC, among which patients with positive TNX displayed a much longer mean survival time than among patients with negative TNX.^30^ However, in recent years, a scarce amount of studies investigating TNX and its specific role and mechanism in CC have been noted. Herein, we also identified the down‐regulation of TNXB in CC cells, which indicated that the overexpression of TNXB could be a positive indicator for CC. Tenascin‐X has been previously reported to affect the activation of the TGF‐β signalling,^31^ with studies suggesting that TGF‐β could potentially interact with the PI3K‐Akt signalling.^32^ In our study, TNXB was found to regulate the PI3K‐Akt signalling pathway.

RETRACTED

Finally, a key observation of the current study revealed that silencing LINC01305 or overexpressed TNXB could inhibit the EMT, migration and invasion of CC cells through inhibiting the activation of the PI3K‐Akt signalling pathway. Previous studies have uncovered that lncRNAs may be up‐regulated or down‐regulated in cancers and operate in an influential fashion in relation to the progression, invasion and metastasis of diverse tumour cells.^33^, ^34^ Chen et  al demonstrated that LINC01512, as an oncogenic lncRNA gene, promotes the proliferation, invasion and migration of lung adenocarcinoma.^35^ Yang et  al indicated that the lncRNA CCHE1 is distinctly up‐regulated in CC tissues, highlighting its pivotal role in CC cell proliferation and invasion by means of elevating proliferating cell nuclear antigen.^8^ Tenascin‐X is primarily involved in the process of organogenesis by supporting cell migration, while the expression of TNXB is higher in malignant mesothelioma (MM) when compared with that of ovarian/peritoneal serous carcinoma.^36^, ^37^ Matrix metalloproteinase 2 and MMP9 have been implicated in the process of metastasis, both of which are capable of regulating the migration and invasion of cancer cells. Furthermore, the levels of MMP2 and MMP9 are significantly increased in a large array of human tumours and are regarded as important prognostic factors in cases of CC.^38^ Matsumoto et  al provided elucidation regarding the tumour metastasis and invasion of grafted melanoma cells, which exhibited enhanced levels in mice with deficient TNX, while the levels of MMP2 and MMP9 increased among TNX‐deficient mice in vivo, the up‐regulation of which is thought to promote melanoma cell invasion and dissemination.^36^ Reports have suggested that LINC00152 inhibition suppresses cell invasion, migration as well as proliferation abilities, while promoting cell apoptosis in non‐small cell lung cancer, which is accompanied by reduced expressions of epidermal growth factor receptor (EGFR), PI3K, Akt, Fibronectin and vimentin proteins, as well as increased P21 protein expression.^39^ PI3K/Akt is a downstream signal transduction pathway of EGFR expression, which is activated through cell cyclin dependent kinase, while P21 works as an inhibitor of that kinase.^40^, ^41^ Reports have correlated down‐regulated E‐cadherin and up‐regulated vimentin with enhanced migration of tumour cells, leading to higher metastatic risk of patients with head and neck squamous cell carcinomas.^42^ EMT represents a biological conversion process of polarized epithelial cells to mesenchymal phenotype, featured by the loss of cell‐cell adhesion, epithelial polarity and the acquisition of migratory and invasive properties.^43^, ^44^ The loss of E‐cadherin is a hallmark of EMT regulated by an array of signalling networks, embracing PI3K/Akt, extracellular, signal‐regulated protein kinases, Smads, mitogen‐activated, protein kinase and RhoB and β‐catenin.^44^, ^45^ Taken together, the aforementioned studies provided support for the conclusion of our study.

In conclusion, the results from this present study proved our hypothesis that LINC01305 silencing inhibited EMT, invasion and migration of CC cells via the inhibition of the PI3K/Akt signalling pathway by targeting TNXB. Hence, we propose that our investigation results may offer a novel therapeutic method for the treatment of CC. However, as LINC01305 remains a relatively recently discovered gene, its role in the treatment of CC and application in other cancers requires future investigation.

RETRACTED

## CONFLICT OF INTEREST

The authors have declared that no competing interests exist.
